This article has been retracted.

# Impacts of lipopolysaccharide on fetal lung developmental maturity and surfactant protein B and surfactant protein C protein expression in gestational diabetes mellitus rats

**DOI:** 10.1080/21655979.2021.2013099

**Published:** 2022-01-09

**Authors:** Yue Gao, Ziwei Zhang, Yan Wang, Dayong Zhou, Jinghua Zhang, Xiaoyu Chen, Xin Li, Qingliang Shao

**Affiliations:** a Department of Neonatal, The Fourth Hospital of Harbin Medical University, Harbin; b Public Affairs Management, Medical University of Tianjin, Tianjin, China; c Rehabilitation Center, The Second Affiliated Hospital of Heilongjiang University of Chinese Medicine, Harbin, China; d Children’s Rehabilitation Center, Heilongjiang Seamen General Hospital, Harbin, China; e Department of Health Care, Harbin City Maternal and Child Health Care Family Planning Service Center, Harbin, China

**Keywords:** Information technology, gdm rats, fetal lung developmental maturity, sp-b and sp-c protein expression

## Abstract

The rise of bioinformatics based on computer medicine provides a new method to reveal the complex biological data. This experiment is to explore the impacts of lipopolysaccharide on fetal lung developmental maturity and expressions of lung surfactant protein B (SP-B) and lung surfactant protein C (SP-C) in rats with gestational diabetes mellitus (GDM), thereby discussing the mechanism of developmental disorders in rats. Forty-eight conceived female rats were experimental subjects. Twenty-eight rats were randomly selected to construct the GDM models. All conceived rats underwent section on the 21st day of pregnancy. The ultrastructure of alveolar type II epithelial cells and the morphology of lung tissue were observed under a microscope. The protein localization and expression of SP-B and SP-C were determined by immunohistochemistry; the protein levels of SP-B and SP-C were determined by Western blot. Blood glucose and body weight of the GDM group were higher than those of the control group; the number of alveoli and alveolar area in the GDM group was lower than those in the control group; the alveolar interval in the GDM group was significantly higher than that in the control group (*P* < 0.05). The average absorbance of SP-B and SP-C in fetal lung tissue was significantly lower in the GDM group than that in the control group (*P* < 0.01). Changes in fetal lung tissue structure of rats were related to SP-B and SP-C, which was one of the main factors that affected the maturation of fetal lung tissue.

## 1. Introduction

With the continuous development of science and technology, computer information technology has been enhanced rapidly and utilized widely in the medical field, which has also become an independent discipline – medical informatics. Reports suggest that the application of computer information technology has improved the cure rate of diseases and prolonged the lifespan of humans. Therefore, it plays a vital role in the medical field, which accelerates the development of the medical field. Moreover, it also has great development prospects in the medical field. Biochip has the advantages of high throughput and rapid measurement. It can produce massive and complex biological information data. However, how to interpret the hybridization information of a large number of gene points on the chip and reveal the life characteristics and laws contained has become the main research content of the application and development of gene chip technology.

One of the common complications in pregnancy is gestational diabetes mellitus (GDM). Fetal lung maturation disorder is one of the common diseases of fetuses born by pregnant women with GDM, who will suffer from respiratory distress syndrome (RDS) [1]. Lung surfactant protein B (SP-B) and lung surfactant protein C (SP-C) are common proteins on the lung surface, which can regulate the alveolar surface tension and also maintain normal breathing to some extent. Studies have found that thyroid transcription factor-1 and multi-line adenoma-like factor-2 regulate the expression of SP-B and SP-C to some extent [2,3]. Pulmonary surfactant is a complex composed of phospholipids and surfactant-specific proteins. Among them, the most biophysically active components are saturated phosphatidylcholine, SP-B and SP-C, which can reduce the tension of the gas-liquid interface to a very low level. Pulmonary surfactant is synthesized by type II alveolar epithelial cells and stored in lamellar bodies for basic secretion or secretion under certain stimulating factors such as β-agonist and lung stretch. Under normal circumstances, the surfactant is swallowed and decomposed by macrophages or recycled to type II cells to synthesize new surfactants or participate in catabolism. Researches have reported that the knockout or deletion of the SP-B and SP-C genes can cause respiratory failure and eventually death [4,5]. Pulmonary infection is a common clinical infectious disease, which usually occurs in the patient after surgery or with lung disease, while timely and effective diagnosis and treatment are extremely important for patients [6]. Lung infection is accompanied by symptoms such as cough, sputum, chest pain, and dyspnea. If the disease is not effectively treated, the patient may die. Pulmonary infections can cause breathing disorders, resulting in abnormal gas exchange, which reduces the concentration of oxygen in the body and increases the concentration of carbon dioxide; eventually, it leads to disorders of physiological metabolism and complications such as acute respiratory failure [7,8].

This exploration aims to investigate the effects of lipopolysaccharide on the development and maturity of fetal lung and the expression of SP-B and SP-C proteins in GDM rats, and then to explore the mechanism of developmental disorder in rats. In this experiment, the GDM rat model is established, the ultrastructure and morphological structure of lung tissue are observed, the protein localization and expression of SP-B and SP-C and their mRNA levels are measured, which provide a basis for clinical treatment of lung diseases.

## 2. Materials and methods

### 2.1. Experimental animal and fetal sampling

Overall, 50 healthy and clean Sprague-Dawley (SD) virgin rats (10 weeks old, with a weight of about 265 g) and 10 male rats were purchased from Laboratory Animal Center. All animals were fed in cages with rodents of national standards. The male and female rats were caged at a 3: 1 ratio overnight. The vaginal smears of female rats were performed early the next morning. If the sperm could be observed under the microscope, it was recorded as the first day of pregnancy. Finally, 48 female rats were conceived. Twenty-eight rats were randomly selected to construct the GDM models, which is the GDM group. The remaining 20 conceived rats were the control group. All rats were given natural illumination and free diets. The room temperature and humidity were controlled at 20–26°C and 40–50%, respectively. The adaptive feeding continued for 2 weeks. The blood glucose levels of conceived rats were tested randomly on the 21st day of pregnancy. Then, the fetal rats were obtained through the cesarean section [9]. This operation must be performed under aseptic conditions. Each fetus was obtained and weighed. There were 120 fetuses in the GDM group and 170 fetuses in the control group. The processes of animals and the experimental procedures were conducted under the Chinese Experimental Animal Protection and Management Regulations and were submitted to the approval of the superior ethics committee. The operation and treatment of animals in this experiment comply with the basic ethical norms of biomedical animal experiments.

### 2.2. Ultrastructure of alveolar type II epithelial cells and observation of lung morphology

Fresh fetal lung tissues were taken from 6 randomly selected fetal rats to observe the ultrastructure of alveolar type II epithelial cells. The tissues were fixed in 2.5% glutaraldehyde (Shandong Pengda Industrial Co., Ltd., China). Then, they were dehydrated in 75%, 80%, 85%, 90%, 95%, and 100% alcohol (Fine Chemical Plant of Economic and Technological Development Zone, China) successively. Next, the tissues were dehydrated again in 70%, 80%, 90%, and 100% acetone (Shandong Zhongji Chemical Co., Ltd., China) successively. Afterward, they were made into paraffin-embedded sections, double-stained with 3% uranium acetate (Xi’an Dingtian Chemical Co., Ltd., China)-lead citrate (Weifang Ruiding Biotechnology Co., Ltd., China), and observed under an electron microscope (OLYMPUS, Japan). Fifty fetal rats were randomly selected from the GDM group and the control group, respectively. The morphology and structure of selected fresh fetal lung tissues were observed. Before observation, the fresh tissues were fixed with 4% formaldehyde (Fine Chemical Plant of Economic and Technological Development Zone, China). Then, the tissues were sequentially dehydrated with 75%, 80%, 85%, 90%, 95%, and 100% alcohol, embedded with paraffin, dewaxed, sectioned, and washed with distilled water for 5 min. Next, tissue sections were stained with Hematoxylin-Eosin (HE) and observed under a microscope (OLYMPUS, Japan).

### 2.3. Immunohistochemistry

The expression of SP-B and SP-C protein in fetal lung tissue was determined by immunohistochemistry. After the fresh fetal lung tissues were embedded and sectioned, the discontinuous sections were randomly selected and blocked with 10% goat serum (Shanghai Beyotime Biotechnology Co., Ltd., China) to block the nonspecific staining. The procedures should strictly follow the immunohistochemistry kit (Wuhan BOSTER Biological Technology Co., Ltd., China). The samples were added with the first antibody (Santa Cruz, USA) at a concentration of 1: 100, incubated at 4°C overnight, added with the second antibody (Wuhan Sanying Co., Ltd., China), incubated at 37°C for 45 min, added with horseradish peroxidase (Western Instrument (Beijing) Technology Co., Ltd., China) labeled streptavidin, incubated for 45 min at 37°C, developed with diaminobenzidine (Chengdu Jiaye Biological Technology Co., Ltd., China), counterstained with hematoxylin (Weifang Ruiding Biotechnology Co., Ltd., China), and observed under an electron microscope.

### 2.4. Western blot

The fresh fetal rat lung tissues were put into a 1 mL EP tube. The protein lysate (TaKaRa, China) and protease inhibitor/phosphatase inhibitor (TaKaRa, China) were prepared at a ratio of 100: 1. The tissues were added with protein lysate, ground, homogenized, stood, and centrifuged. Then, the supernatant was removed. The protein concentration was detected by the bicinchoninic acid (BCA) method, and the sodium salt-polyacrylamide gel electrophoresis (SDS-PAGE) (Sigma, USA) was performed. After the gel electrophoresis was completed, the location of the desired protein molecules was found. The gel was cut and then put in a cold electro-transfer solution. The polyvinylidene fluoride (PVDF) membrane that had been soaked in methanol and buffer was marked. The filter paper was immersed in the electro-transfer solution. The film was transferred in the order of filter paper/gel/PVDF membrane (BOSTER Biological Technology Co., Ltd., China)/filter paper. Then, the transferred membrane was washed with Tris-HCl buffered salt solution + Tween (TBST) (Shanghai Tuhe Industrial Co., Ltd., China). The transferred PVDF membrane was blocked with the prepared skim milk powder for 2 h, incubated with the first antibody (Rabbit anti mouse fibroblast growth factor-7 polyclonal antibody) and the second antibody (biomarker Goat anti rabbit secondary antibody) (CST, USA), and washed with TBST solution to develop the color. The gray value was calculated.

### 2.5. Fluorescence real-time quantitative polymerase chain reaction (RT-qPCR)

Overall, 100 mg fresh fetal lung tissue was taken, the total RNA was extracted from the cells, and the mass was determined to be 500 ng after measuring the RNA concentration. The required reverse transcription volume was obtained, and the reverse transcription reaction was strictly performed under the instructions of the SYBR Premix Ex Taq reverse transcription kit (TAKARA, Japan). The reaction system was as follows: 2 μL cDNA, 10 μL SYBRII, 0.4 μL upstream primer, and 8.0 μL ultra-pure water. With β-actin as an internal reference, the reaction was performed under the following conditions: pre-denaturation at 95°C for 30 s, reaction at 95°C for 5 s, reaction at 60°C for 30 s, repetition of the above for 40 cycles, reaction at 94°C for 90 s, and extension at 60°C for 180 s. RT-qPCR was used to detect the relative mRNA expression of proinflammatory cytokines interleukin-11β (IL-1β) and tumor necrosis factor-α (TNF-α) in fetal lung and fetal membranes.

### 2.6. Data analysis

*P* < 0.05 indicated that the difference is statistically significant. SPSS software was used for analysis. Kruskal-Wallis test was used for pathological inflammation grade comparison, and Mann-Whitney test was used for multiple comparisons among groups. The measurement data of normal distribution were expressed by mean ± standard deviation. The analysis of variance was used for inter-group comparison, and the q-test was used for pairwise comparison. If the variance was uneven, Dunnett’s T3 method was used. *P* < 0.05 indicated a significant difference, and *P* < 0.01 indicated a notably significant difference.

## 3. Results and analysis

GDM is a common disease in women during pregnancy, which is easy to lead to various adverse pregnancy outcomes. It will not only bring serious health risks to pregnant women, but also make future generations face great health challenges. Prenatal glucocorticoid is the standard treatment for promoting fetal lung maturation in preterm infants. Through the synchronous induction and inhibition of multiple genes, the lipid and surfactant protein on the lung surface are finally increased, and the lung interstitium is thinned to increase the potential alveolar cavity, so as to promote lung maturation. The effects of lipopolysaccharide on the developmental maturity and the expression of SP-B and SP-C in the fetal lung of GDM rats are studied, so as to explore the mechanism of developmental disorder in rats.

### 3.1. Blood glucose of conceived rats and the body weight of fetuses

Figure 1 displayed the blood glucose of conceived rats and the body weight of fetuses. Compared with the conceived rats in the control group, the conceived rats in the GDM group had polydipsia, polyphagia, and polyuria. On the 21st day of pregnancy, the blood glucose level in the GDM group (26 mmol/L) was higher than that in the control group (5 mmol/L). When the fetal rats were taken through cesarean section, the amniotic fluid of the conceived rats in the GDM group was thick, clear, and brushable. The average number of fetal rats delivered by the conceived rats in the GDM group was lower than that of the control group, which were 6 and 11, respectively. The average body weight of the fetal rats after delivery in the GDM group was higher than that in the control group, which was 5.5 g and 5.1 g, respectively. The differences between these indicators of the two groups were not statistically significant.

**Figure 1.** Blood glucose of conceived rats and body weight of fetuses.

### 3.2. Inflammatory pathological changes of the fetal lung, fetal membrane and placenta in rats

A scoring system was established to assess the histological severity of inflammation in HE sections of fetal lung, placenta and fetal membrane (amnion). The score of fetal pneumonia from 0 to 4 indicated that the fetal lung had changed from ‘no pathological manifestation’ to ‘destruction of normal lung tissue structure and necrosis of lung parenchyma’. The score of umbilical vasculitis from 0 to 4 indicated that the blood vessels had changed from ‘no pathological manifestations’ to ‘nuclear fragmentation, nuclear concentration or nuclear lysis under the vascular endothelium’. The score of chorioamnionitis from 0 to 4 indicated ‘no pathological manifestations’ to ‘degeneration or abscission of amniotic epithelial cells’. Figure 2, Figure 3 and Figure 4 were representatives of the HE section of the inflammatory score of the fetal lung, placenta and fetal membrane. Multiple comparisons of histopathological scores of rats in two groups showed that the inflammation scores of the GDM group were significantly higher than those of the control group.

**Figure 2.** The representative figure of inflammation score of fetal lung tissue in rats (a: control group; b: GDM group).

**Figure 3.** The representative figure of inflammation score of rat fetal membrane (amnion) (a: control group; b: GDM group).

**Figure 4.** The representative figure of inflammation score of rat placenta (a: control group; b: GDM group).

### 3.3. Ultrastructure of alveolar type II epithelial cells

Figure 5 presented the ultrastructure of fetal rat alveolar type II epithelial cells. Observation under the electron microscope showed that the villi on the surface of alveolar type II epithelial cells in the control group of fetuses were thin, long, and regular in shape. There were massive fetal lung lamellar corpuscles, the hierarchical structure was visible, and the staining was deep. There were multiple organelles in the cytoplasm; besides, there were no swelling or fat particles in the mitochondria. In the GDM group, the villi on the surface of the alveolar type II epithelial cells of the fetal rats were thick, short and irregular in shape; the number of lamellar bodies in the fetal lung was small, and the staining was light. There were fewer cytoplasmic organelles, increased glycogen, and fat particles. The rupture of the basement membrane was discontinuous and uneven in thickness.

**Figure 5.** Ultrastructure of fetal rat alveolar type II epithelial cells (a-c: The control group; d-f: The GDM group).

### 3.4. Morphology and structure of fetal lung tissue

Figure 6 revealed the morphology and structure of the fetal rat lung tissue. Figure 6 suggested that under the electron microscope, the alveolar structure of the fetal rats in the control group was regular, uniform in size and space, with little knot tissue, no edema, increased inflammation, fibrous tissue hyperplasia, and alveolar cavity exudation. In the GDM group, the alveoli were fewer and irregularly arranged. The alveolar area was decreased, the alveolar cavity structure was increased, the alveolar space was uneven, and nodal tissue was increased. Figure 6 revealed that in the control group, the average number and area of the alveolar were significantly higher than those of the GDM group (*P* < 0.01), while the alveolar interval was significantly lower in the control group than that of the GDM group (*P* < 0.01).

**Figure 6.** Morphology and structure of fetal lung tissue (a, b: Morphology and structure of fetal lung tissue; c: Average number of alveoli and alveolar space; d: Average area of alveoli; *P < 0.01).

### 3.5. SP-B and SP-C protein localization and expression

Figure 7 showed the protein localization and expression results of SP-B and SP-C in fetal rat lung tissue. Figure 7 suggested that the protein expression of the control group was continuous, while that of the GDM group was discontinuous. Figure 7 revealed that the absorbance of SP-B and SP-C in the GDM group was significantly lower than that of the control group (*P* < 0.01).

**Figure 7.** SP-B and SP-C protein localization and expression (A, B: The control group; c, d: The GDM group; E: The absorbance; * *P* < 0.01).

### 3.6. Protein and mRNA levels of SP-B and SP-C

Figure 8 presented the protein and mRNA levels of SP-B and SP-C. Figure 8 showed that the protein levels of SP-B and SP-C in the GDM group were significantly lower than those in the control group (*P* < 0.01). Figure 8 suggested that the mRNA levels of SP-B and SP-C were also significantly lower in the GDM group than those in the control group (P < 0.01). Figure 9 presented the results of RT-qPCR for SP-B and SP-C protein mRNA levels in the lung tissues of the two groups of rats.

**Figure 8.** The protein and mRNA levels of SP-B and SP-C (a: The protein level; b: The mRNA level; *P < 0.01).

**Figure 9.** RT-qPCR results of SP-B and SP-C protein mRNA levels in lung tissue of two groups of rats.

### 3.7. Relative mRNA expression of IL-1β and TNF-α in fetal lung and fetal membrane of rats

Figure 10 and Figure 11 showed the relative mRNAs expression of IL-1β and TNF-α in fetal lung and fetal membrane of the two groups of rats. It revealed that compared with the control group, the expression of proinflammatory cytokines IL-1β and TNF-α in the fetal lung tissue and fetal membrane tissue of the GDM group was significantly higher. There was a statistical difference between the two groups (*P* < 0.01).

**Figure 10.** The comparison of the IL-1β mRNAs expression in fetal lung and fetal membrane of rats in two groups (* compared with the control group, *P* < 0.01).

**Figure 11.** The comparison of the TNF-α mRNAs expression in fetal lung and fetal membrane of rats in two groups (* compared with the control group, *P* < 0.01).

## 4. Discussions

From the perspective of the fetus, GDM will cause problems such as macrosomia, shoulder dystocia, premature delivery and hypoxia, which greatly increases the production time. Moreover, the risk of fetal complications such as hypoglycemia, hyperbilirubinemia and pneumonia will be higher than that of normal fetuses, even including the probability of developing type 1 diabetes. Research has found that GDM has a certain effect on the development of fetal lung tissue [10]. If the blood glucose level of pregnant women with GDM is high, the blood glucose will reach the fetus through the placenta; as a consequence, the fetal insulin level will rise and hyperinsulinemia will occur, which will have an inhibitory effect on the synthesis and release of lung surfactant, leading to the prolonged maturity of the fetal lung; also, the occurrence of RDS will increase 1 month after the neonate is born [11]. Pulmonary surfactants are composed of SP and phospholipids secreted and synthesized by alveolar type II epithelial cells. They form a water-insoluble phospholipid-protein layer that consists of lowering alveolar surface tension, which maintains normal breathing [12,13]. Some studies have found that SP-B and SP-C are the main hydrophobins. When the SP-B gene is silenced, severe respiratory failure symptoms will occur and eventually lead to death [14,15]. Pulmonary surfactant is a complex composed of phospholipids and surfactant-specific proteins. Among them, the most biophysically active components are saturated phosphatidylcholine, SP-B and SP-C, which can reduce the tension of the gas-liquid interface to a very low level. Besides, the deletion of the SP-B gene is a crucial factor leading to the occurrence of RDS in 1-month-old neonates. Research reveals that after the SP-C gene is knocked out, the mice do not develop acute respiratory failure; however, soon, multiple lung diseases occur, which eventually leads to death [16,17]. The SP-B and SP-C genes are affected by multiple factors, such as hormone levels, development, and various nuclear protein factors. A study suggests that the development of the lungs of rats is similar to humans. The development of the lungs of fetuses at 21 days of gestational age can fully reflect the characteristics and developmental symptoms of fetal lung function during pregnancy [18,19].

The lung structure of the fetuses taken at 21 days of pregnancy was studied by building the GDM pregnant rat models. Observation under the electron microscope revealed that the villi on the surface of the alveolar type II epithelial cells of the control group were elongated and regular in shape, with massive lamellar bodies, clear hierarchical structure, and deep staining. There were also multiple cytoplasmic organelles, no swelling of mitochondria, and no fat particles. In the GDM group, the villi on the surface of the alveolar type II epithelial cells of the fetal rat were thick, short, and irregular. There were fewer cytoplasmic organelles, increased glycogen, and fat particles. The rupture of the basement membrane was discontinuous and uneven in thickness. These results were consistent with the results of previous research [20,21]. The alveoli of fetal rats in the GDM group were fewer and irregularly arranged. The alveolar area was decreased, the alveolar cavity structure was increased, the alveolar space was uneven, and nodal tissue was increased. No transparent substance was seen, which was probably because it was more common in rats that died after birth. Through RT-qPCR and Western blot, it was found that the protein and mRNA levels of SP-B and SP-C in the fetal lung of the GDM group were lower than those of the control group.

This experiment found that changes in fetal lung tissue structure of rats were related to SP-B and SP-C, which was one of the main factors affecting the maturation of fetal lung tissue.

## 5. Conclusions

This experiment explored the impacts of lipopolysaccharide on fetal lung developmental maturity and expressions of SP-B and SP-C in GDM rats. The results showed that blood glucose and body weight in the GDM group were higher than those in the control group; the number of alveoli and alveolar area in the GDM group was lower than those in the control group; the alveolar interval in the GDM group was significantly higher than that in the control group. The average absorbance of SP-B and SP-C in fetal lung tissue was significantly lower in the GDM group than that in the control group. The SP-B and SP-C protein levels in fetal lung tissue were significantly lower in the GDM group than those in the control group. Therefore, changes in fetal lung tissue structure of rats were related to SP-B and SP-C, which was one of the main factors that affected the maturation of fetal lung tissue.
